# Computer Navigation-Aided Excision of Proximal Femoral Osteochondroma: Surgical Technique

**DOI:** 10.1155/2022/7635945

**Published:** 2022-05-31

**Authors:** Yang Sun, Chun Ming Chan, Feng Yu, Yuan Li, Xiaohui Niu

**Affiliations:** ^1^Department of Orthopedic Oncology, Beijing Ji Shui Tan Hospital, No. 31 Xin jie kou Dong Jie, Xi Cheng District, Beijing 100035, China; ^2^National University Hospital, Singapore

## Abstract

**Purpose:**

Symptomatic osteochondroma of the proximal femur necessitates a surgical excision. The purpose of this study was to describe a novel technique of computer navigation-aided excision for osteochondromata of the proximal femur. Outcomes of this technique are also presented.

**Methods:**

A total of 13 patients underwent computer navigation-aided excision of osteochondromata of the proximal femur from February 2012 to August 2016 in our institution. They were enrolled in this study. OrthoMap 3D (Stryker Orthopaedics, Mahwah, NJ, USA), a commercially available navigation software system, was used to merge computed tomography images of the proximal femur with an osteochondromata with the image of a normal proximal femur. Using the normal proximal femur as a template, intended resection margins for the proximal femur with osteochondromata were planned and then executed using intraoperative navigation guidance. Patients were followed up clinically and radiographically. The physical and mental health of patients was assessed with the Musculoskeletal Tumor Society (MSTS) score.

**Results:**

Eight patients had isolated exostoses. Five patients had tumors associated with multiple hereditary exostoses. For tumors projecting posteriorly or posteromedially, a posterolateral approach was used. For tumors projecting anteriorly or medially, an anterior approach was used. Prophylactic fixation was performed in four patients who required an anterior approach. The mean duration of the surgery was 189 minutes. There were no intraoperative fractures or postoperative complications. A secondary procedure was not needed for any case. The mean MSTS score at a mean follow-up of 17 months was 28.6 (maximum MSTS score: 30).

**Conclusions:**

This is the first study to report a novel application of computer navigation for aiding the excision of osteochondromata of the proximal femur. It demonstrated favorable postoperative functional scores with a low rate of complications. The applicability, safety, and efficacy of this technique were demonstrated. It is particularly useful for resections involving large tumors that can obscure anatomical landmarks and for patients with associated proximal femoral deformity.

## 1. Introduction

Osteochondroma is a benign bone tumor that usually affects the pelvis, knee, tibia, and femur [1]. However, it can also occur as a solitary tumor [2]. Multiple osteochondromata, also known as multiple hereditary exostoses (MHE), can also occur [3]. Most osteochondroma patients do not show sufficient symptoms that necessitate surgery. Spontaneous regression of osteochondroma has been reported [4, 5]. For patients suffering from significant symptoms and those who show malignant transformation, surgical removal is needed [6, 7]. Osteochondroma that occurs in the proximal femur can show symptoms such as pain [8, 9], impingement [10], and sciatica secondary to nerve compression [11, 12]. Osteochondroma in the proximal femur can also lead to abnormal proximal femur development and deformities (including acetabular dysplasia and coxa valgus) [13, 14]. Resecting the osteochondroma of the proximal femur is different from resecting other osteochondromata (i.e., osteochondroma found in places other than the proximal femur). First, an osteochondroma of the proximal femur has close proximity to vital structures, making it challenging to obtain adequate exposure. Second, the femoral neck is subjected to high stress and high load. Third, prophylactic fixation is frequently needed because the structural integrity might be affected when resecting an osteochondroma of the proximal femur. The objective of this study was to describe a technique of using computer navigation to aid in the resection of osteochondroma in the proximal femur so that adequate tumor removal could be achieved while the native bone stock. Outcomes of patients using this procedure are also presented.

## 2. Materials and Methods

From February 2012 to August 2016, patients who underwent osteochondroma resection in the proximal femur aided by computer navigation were identified. This study was approved by the Medical Ethics Committee of the Beijing Ji Shui Tan Hospital (BJST2021-52). Prior to study inclusion, patients provided informed consent. Inclusion criteria are as follows: (1) osteochondroma of proximal femur; (2) the tumor was removed by computer-aided navigation technology during operation; and (3) the medical records and follow-up data are complete, and the follow-up time is 6 months or more. Hospital records of these patients were reviewed. A total of 13 patients with a minimum follow-up of six months were found to be eligible for this study. The mean follow-up was 17 months (range, 7-60 months). There were seven males and six females. The age of the patients ranged from 16 to 49 years (mean age: 29.9 years). Radiographic imaging and computed tomography were performed before surgery. Follow-up points included 3 months, 6 months, 12 months, 18 months, and 24 months. During follow-up visits, radiographic imaging was performed. The Musculoskeletal Tumor Society (MSTS) score [15] was used to assess their functional outcomes.

### 2.1. Preoperative Planning and Surgical Technique

The preoperative plan created for each patient in this series was the same. A commercially available navigation software system (OrthoMap 3D, Stryker Orthopaedics, Mahwah, NJ, USA) was used to create the preoperative plan. It was also used for the intraoperative computer navigation.

For each patient, a gender- and size-matched normal proximal femur was identified from our institution's image database. Specifically, the parameters used for the two femora were femoral head diameter, femur neck diameter, proximal femur diaphyseal diameter, and femoral neck angle. Computerized tomography (CT) images of the patient and the normal femur were uploaded onto the navigation software. These two images were then merged. Merged images were used to confirm whether there was a satisfactory match of the proximal femoral geometry. Intended resection margins were then drawn on CT images of patients' proximal femora using the normal proximal femur as a template. This means of templating was intended to maximize bone preservation. The time required for preoperative planning was estimated to be between 60 and 90 minutes for each case.

The approach to access the proximal femur was chosen by the attending surgeon for each patient according to the orientation of the osteochondroma. Once adequate exposure was obtained, tracking markers were secured to the femur distal to the operative site using transosseous half pins. Registration of the patient's femoral anatomy on the navigation system was performed automatically using images acquired with an isocentric C-arm system (Arcadis Orbic, Siemens AG, Erlangen, Germany) during an intraoperative CT scan. Using a navigation stylus, preoperative margins were marked on the bone, and the appropriate axis for performing the resection was confirmed. Osteotomies were then performed with a combination of osteotomes and high-speed burr. The navigation stylus was then used to confirm that the resection performed matched the preoperative plan. In contrast to performing osteotomies while resecting malignant bone tumors, care was taken to avoid overresection (i.e., resecting more normal bone for a wider margin). When performing osteotomies, underresection was preferred to overresection. When necessary, refinement of the resection was performed using a burr when underresection was noted on the navigation system to verify that the resection matched the preoperative plan. Once resections were complete, the passive range of motion of the hip was assessed to confirm the lack of an overt impingement. The attending surgeon decided whether a prophylactic fixation was needed. Patients were allowed to perform partial-weight-bearing ambulation in the immediate postoperative period and full-weight bearing after the first month. Range of motion exercises was initiated at two weeks postoperatively.

## 3. Results

The clinical data of 13 patients included in this study are summarized in Table 1. In the present study, all patients showed symptoms of pain and impingement. Two patients also had sciatica. Eight patients had isolated exostoses. Five patients had MHE (Table 1). Tumors projected posteromedially or posteriorly in nine patients. For these patients, the resection was performed with a posterolateral approach. Figures 1 and 2 show the operation of Cases 6 and 4, respectively.

**Case 1 .**

The pelvic radiographs showed that the lesion was located in the medial side of the proximal right femur (Figure 1(a)). Through the intraoperative application of computer navigation-aided resection, the morphology of the proximal femur was simultaneously displayed on the transverse, coronal, sagittal, and three-dimensional reconstruction images of CT images (Figure 1(b)). The patient exposed the tumor through the posterolateral approach (Figure 1(c)) and then marked the boundary of the osteotomy under the guidance of a stylus (Figure 1(d)), and the tumor was removed.  Figure 1(e) shows the morphology of the proximal femur after tumor resection.

**Case 2 .**

Figures 2(a) and 2(b) show the patient's preoperative frontal and lateral radiographs. Intraoperative axial CT images are shown in Figure 2(c), in which the designed osteotomy boundary is marked in yellow. As seen in Figure 2(d), the postoperative axial CT image showed that the osteotomy boundary was consistent with the preoperative design.

Four patients had tumors based medially or anteriorly. For these patients, resection was performed with the Smith-Petersen approach, also known as an anterior approach. Prophylactic fixation was performed for four patients. Of these four patients, three received a sliding hip screw, and one received nailing intramedullary. Tumors in these four patients were accessed with an anterior approach. For nailing and plating, an incision was performed laterally. The duration of the surgery ranged from 120 minutes to 285 minutes (mean: 189 minutes). There were no intraoperative fractures. Complications were not observed either. No case needed a secondary procedure that was unplanned. No patient was unsatisfied with the result of the surgery. At the last follow-up, MSTS score ranged from 27 to 30, with a mean score of 28.6. The maximum possible MSTS score was 30.

## 4. Discussion

Resecting osteochondroma and other tumors in the proximal femur is challenging due to the location. It is of paramount importance to obtain adequate exposure. To provide surgical access to this location, a variety of approaches have been reported, including the posterolateral approach [8, 10, 11], the Smith-Petersen approach (also known as the anterior approach) [16], the medial Ludloff approach [17], and the digastric approach [18] with accompanying hip dislocation. To facilitate tumor removal, it is obviously necessary to permit tumor visualization. It is also necessary to achieve adequate exposure so that surgeons can avoid damaging the proximal femur during surgery. The medial proximal femur is a biomechanically important structure [19]. Femoral neck fractures as complications after resecting osteochondroma at this location have been reported [16, 20]. In the present study, patients underwent resection with either a posterolateral approach or an anterior approach aided by computer navigation for confirmation of appropriate axes.

As a bridge connecting the femoral head and femoral shaft, the femoral neck also undertakes the power transmission between the pelvis and lower limbs, so it is also a part with relatively large stress. Due to its deep anatomical position, it is not easy to be exposed by surgery. Therefore, the osteochondroma of the femoral neck may have the problem of insufficient or excessive resection in traditional resection. Incomplete surgical resection of osteochondroma will increase the risk of osteochondroma recurrence. Computer-aided navigation has several advantages for orthopaedic oncology surgeries [21]. For example, when operating at an anatomical site that is hard to access, it can be used to provide extra confirmation. It can guide the performance of complex three-dimensional osteotomies. It can also improve the precision of the performance of osteotomies [22]. Precision is a prerequisite to achieving satisfactory surgical margins while preserving vital structures. Using a computer-aided navigation system, excessive removal of vital bone around the medial femoral neck was minimized in the present study. When tumors had significantly caused distortions anatomically and resulted in few anatomic landmarks, the computer-aided navigation system guided osteotomies. In the present study, two patients had femoral neck tumors without calcar femorale involvement. For these two patients, the computer-aided navigation system allowed us to perform the excision while minimizing bone removal, thus avoiding prophylactic fixation. When approaching a medially based tumor, an anterior approach does not provide ample exposure as a digastric approach. It could provide a direct exposure as a Ludloff approach either. However, since all orthopaedic surgeons are familiar with an anterior approach, utilizing a computer-aided navigation system can help surgeons perform osteotomies accurately.

For patients with femoroacetabular impingement (FAI), computer can be used to model dynamic impingement and hip movements during preoperative planning [23, 24]. In those studies, considering impingement and dynamic factors, hip range of motion was predicted accurately after osteoplasty. The present study was performed based on the hypothesis that restoring the proximal femur's normal anatomy could improve pain caused by bony impingement. Although computer modelling is more comprehensive than our technique, our method has an advantage in that it uses a computer navigation system that is commercially available.

In conclusion, this study describes a novel application of a computer-aided navigation system for aiding the resection of osteochondroma of the proximal femur. It can help surgeons perform adequate tumor removal while minimizing excessive removal of bone that is structurally important.

## Figures and Tables

**Figure 1:** Preoperative planning and intraoperative pictures of patient 6. (a) Preoperative AP pelvic radiographs. (b) Computer screenshot during intraoperative navigation depicting axial CT image, coronal, and sagittal reconstructions. Preoperative plan for osteotomy marked in magenta. The green line depicts intraoperative position of navigation stylus. The yellow circles depict the pre-233 operative plan for resection margin. (c) Exposure via a posterolateral approach. (d) Osteotomy plane marked using a stylus. (e) Femoral neck following tumor resection.

**Figure 2:** Imaging studies of patient 4. (a) AP and (b) lateral preoperative radiographs. (c) Axial CT with resection plan marked in yellow. (d) Postoperative axial CT.

**Table 1:** Clinical data of 13 patients included in this study.

Case	Age	Sex	Side	MHE?	Site of tumor	Location of pain/presenting symptoms	Approach	Prophylactic fixation	Complications	Follow-up (as of March 2015)	MSTS score
1	38	M	L	No	Posteromedial	Gluteus	Posterolateral	None	None	27	30
2	25	F	L	No	Medial	Thigh	Anterior	Nail	None	17	27
3	29	M	L	No	Posteromedial	Inguinal	Posterolateral	None	None	12	28
4	25	F	L	No	Posterior	Sciatica	Posterolateral	None	None	12	30
5	18	M	L	Yes	Anteromedial	Thigh	Anterior	DHS	None	9	28
6	19	F	R	No	Medial	Inguinal	Anterior	DHS	None	8	30
7	24	F	L	Yes	Anterior	Inguinal	Anterior	DHS	None	7	27
8	49	M	L	Yes	Posterior	Inguinal	Posterolateral	None	None	12	28
9	37	M	R	Yes	Posterior	Sciatica	Posterolateral	None	None	24	28
10	55	F	L	Yes	Posteromedial	Impingement	Posterolateral	None	None	12	29
11	38	F	L	No	Posterior	Impingement	Posterolateral	None	None	12	30
12	16	M	L	No	Medial	Inguinal	Posterolateral	None	None	60	27
13	16	M	R	No	Medial	Inguinal	Posterolateral	None	None	9	30

## Data Availability

The data used to support the findings of this study are available from the corresponding author upon request.

## References

[1] Galanis V., Georgiadi K., Balomenos V., Tsoucalas G., Thomaidis V., Fiska A. (2020). Osteochondroma of the talus in a 19-year-old female: a case report and review of the literature. *The Foot*.

[2] Ventura-Parellada C., Subirà-I-Álvarez T., Martínez-Ruiz A. (2021). Osteocondroma solitario en el hueso pisiforme con artrosis piso-piramidal. A proposito de un caso. *Revista Española de Cirugía Ortopédica y Traumatología (English Edition)*.

[3] DuBose C. O. (2016). Multiple hereditary exostoses. *Radiologic Technology*.

[4] Passanise A. M., Mehlman C. T., Wall E. J., Dieterle J. P. (2011). Radiographic evidence of regression of a solitary osteochondroma: a report of 4 cases and a literature review. *Journal of Pediatric Orthopedics*.

[5] Le H. M., Schwartz R. B., Corrado G. (2021). Femoral injury over the site of spontaneous regression of an osteochondroma in a teenage athlete. *Current Sports Medicine Reports*.

[6] Ahmed A. R., Tan T. S., Unni K. K., Collins M. S., Wenger D. E., Sim F. H. (2003). Secondary chondrosarcoma in osteochondroma: report of 107 patients. *Clinical Orthopaedics and Related Research*.

[7] Staals E. L., Bacchini P., Mercuri M., Bertoni F. (2007). Dedifferentiated chondrosarcomas arising in preexisting osteochondromas. *The Journal of Bone and Joint Surgery. American Volume*.

[8] Kanauchi T., Suganuma J., Kawasaki T. (2012). Fracture of an osteochondroma of the femoral neck caused by impingement against the ischium. *Orthopedics*.

[9] Muzaffar N., Bashir N., Baba A., Ahmad A., Ahmad N. (2012). Isolated osteochondroma of the femoral neck presenting as hip and leg pain. A case study. *Ortopedia, Traumatologia, Rehabilitacja*.

[10] Hussain W., Avedian R., Terry M., Peabody T. (2010). Solitary osteochondroma of the proximal femur and femoral acetabular impingement. *Orthopedics*.

[11] Yu K., Meehan J. P., Fritz A., Jamali A. A. (2010). Osteochondroma of the femoral neck: a rare cause of sciatic nerve compression. *Orthopedics*.

[12] Turan Ilica A., Yasar E., Tuba Sanal H., Duran C., Guvenc I. (2008). Sciatic nerve compression due to femoral neck osteochondroma: MDCT and MR findings. *Clinical Rheumatology*.

[13] Felix N. A., Mazur J. M., Loveless E. A. (2000). Acetabular dysplasia associated with hereditary multiple exostoses: a case report. *Journal of Bone and Joint Surgery (British)*.

[14] Makhdom A. M., Jiang F., Hamdy R. C., Benaroch T. E., Lavigne M., Saran N. (2014). Hip joint osteochondroma: systematic review of the literature and report of three further cases. *Advances in Orthopedics*.

[15] Enneking W. F., Dunham W., Gebhardt M. C., Malawar M., Pritchard D. J. (1993). A system for the functional evaluation of reconstructive procedures after surgical treatment of tumors of the musculoskeletal system. *Clinical Orthopaedics and Related Research*.

[16] Ramos-Pascua L. R., Sánchez-Herráez S., Alonso-Barrio J. A., Alonso-León A. (2012). Solitary proximal end of femur osteochondroma. An indication and result of the en bloc resection without hip luxation. *Revista Española de Cirugía Ortopédica y Traumatología*.

[17] Chana-Rodríguez F., López-Capapé D., Rojo-Manaute J. (2011). Ludloff approach for osteochondroma in the lesser trochanter in a young middle-distance runner. *European Orthopaedics and Traumatology*.

[18] Li M., Luettringhaus T., Walker K. R., Cole P. A. (2012). Operative treatment of femoral neck osteochondroma through a digastric approach in a pediatric patient. *Journal of Pediatric Orthopaedics. Part B*.

[19] Stiehl J. B., Jacobson D., Carrera G. (2007). Morphological analysis of the proximal femur using quantitative computed tomography. *International Orthopaedics*.

[20] Bottner F., Rodl R., Kordish I., Winklemann W., Gosheger G., Lindner N. (2003). Surgical treatment of symptomatic osteochondroma. A three- to eight-year follow-up study. *Journal of Bone and Joint Surgery. British Volume (London)*.

[21] Wong K. C., Kumta S. M. (2014). Use of computer navigation in orthopedic oncology. *Current Surgery Reports*.

[22] Ritacco L. E., Milano F. E., Farfalli G. L., Ayerza M. A., Muscolo D. L., Aponte-Tinao L. A. (2013). Accuracy of 3-D planning and navigation in bone tumor resection. *Orthopedics*.

[23] Bedi A., Dolan M., Magennis E., Lipman J., Buly R., Kelly B. T. (2012). Computer-assisted modeling of osseous impingement and resection in femoroacetabular impingement. *Arthroscopy*.

[24] Zhang Y., Wen L., Zhang J., Yan G., Zhou Y., Huang B. (2017). Three-dimensional printing and computer navigation assisted hemipelvectomy for en bloc resection of osteochondroma: a case report. *Medicine*.

[25] Yang S., Chan C., Niu X. (2018). Proximal femoral osteochondroma excision aided by computer navigation: surgical technique and case series. *The 18th Annual Meeting of the International Society for Computer Assisted Orthopaedic Surgery*.

